The article "Accurate Identification of Antioxidant Proteins Based on a Combination of Machine Learning Techniques and Hidden Markov Model Profiles" was published in 2021. Journal: Comput Math Methods Med.

# Accurate Identification of Antioxidant Proteins Based on a Combination of Machine Learning Techniques and Hidden Markov Model Profiles

**DOI:** 10.1155/2021/5770981

**Published:** 2021-08-07

**Authors:** Zhehan Shen, Taigang Liu, Ting Xu

**Affiliations:** College of Information Technology, Shanghai Ocean University, Shanghai 201306, China

## Abstract

Antioxidant proteins (AOPs) play important roles in the management and prevention of several human diseases due to their ability to neutralize excess free radicals. However, the identification of AOPs by using wet-lab experimental techniques is often time-consuming and expensive. In this study, we proposed an accurate computational model, called AOP-HMM, to predict AOPs by extracting discriminatory evolutionary features from hidden Markov model (HMM) profiles. First, auto cross-covariance (ACC) variables were applied to transform the HMM profiles into fixed-length feature vectors. Then, we performed the analysis of variance (ANOVA) method to reduce the dimensionality of the raw feature space. Finally, a support vector machine (SVM) classifier was adopted to conduct the prediction of AOPs. To comprehensively evaluate the performance of the proposed AOP-HMM model, the 10-fold cross-validation (CV), the jackknife CV, and the independent test were carried out on two widely used benchmark datasets. The experimental results demonstrated that AOP-HMM outperformed most of the existing methods and could be used to quickly annotate AOPs and guide the experimental process.

## 1. Introduction

A free radical is an atom, molecule, or ion that has an unpaired valence electron, making it highly reactive with other molecules [1]. Reactive oxygen species (ROS) are composed of oxygen-containing free radicals and play important roles in cell signalling and homeostasis [2]. Typically, ROS are present at low and stationary levels in normal cells, involved in a variety of biochemical processes [3]. However, once the organisms suffer from environmental stresses, ROS levels can increase dramatically in the cells, resulting in significant damage to cell structures [2]. Cumulatively, this may lead to a pathological condition known as oxidative stress. In humans, oxidative stress is thought to be involved in the development of several diseases such as ADHD [4], cancer [5], Parkinson [6], Alzheimer [7], and heart failure [8]. Fortunately, cells have evolved defense mechanisms (called antioxidant systems) to keep a check on the generation of ROS and effectively resist the damages caused by ROS [9]. An antioxidant protein (AOP), also known as the free radical scavenger, is a substance that can significantly inhibit oxidation by donating its own electron to ROS and thus neutralize the adverse effects of excess free radicals [10]. The increasing studies have demonstrated that AOPs can promote the immune defense and reduce the hazard of human diseases caused by oxidative stress [11]. Given the importance of AOPs, it has become one of the hot research topics to accurately predict AOPs in protein science. However, due to the complexity of antioxidant mechanisms, it is often time-consuming and laborious to identify AOPs through biochemical experiments [12]. With the huge growth of protein sequences in the last decade, there is an urgent need to develop computational models for the accurate annotation of AOPs based on sequence data only.

The article "Accurate Identification of Antioxidant Proteins Based on a Combination of Machine Learning Techniques and Hidden Markov Model Profiles" was published in 2021. Journal: Comput Math Methods Med.

From the viewpoint of machine learning, identification of AOPs is usually described as a binary classification problem. In recent years, numerous computational methods have been developed to address this problem [12], which mainly focus on two aspects: (1) the feature encoding schemes of protein sequences and (2) the design of classification algorithms. For instance, Fernández-Blanco et al. reported the first machine learning model for the prediction of AOPs by combining the random forest (RF) algorithm and star graph topological indices [13]. However, protein sequences in their dataset shared high sequence similarities, which may lead to the overestimation of predictive performance [14]. Then, Feng et al. constructed a reliable benchmark dataset by removing these redundant protein sequences with the sequence similarity higher than 60% and developed a Naïve Bayes-based model to predict AOPs by using amino acid composition (AAC) and dipeptide composition (DPC) [14]. Unfortunately, the proposed model achieved a relatively low accuracy (Acc) of 66.88% in the jackknife test [14]. Later, Feng et al. adopted a support vector machine (SVM) classifier to improve the prediction of AOPs based on the optimal 3-gap dipeptides obtained by using the analysis of variance (ANOVA) [15]. The overall Acc reached 74.79% on the same dataset [15]. Almost simultaneously, Zhang et al. put forward an RF-based method to distinguish AOPs from non-AOPs by incorporating *g*-gap dipeptide compositions and the position-specific scoring matrix (PSSM) [16]. Their model showed an excellent Acc of 80.7% when tested on an independent dataset [16]. Subsequently, Zhang et al. presented an ensemble classifier to further enhance the predictive performance of AOPs with hybrid features, including secondary structure information (SSI), PSSM, relative solvent accessibility (RSA), and composition, transition, and distribution (CTD) [17]. The ensemble model achieved a balanced performance with a sensitivity (Sen) of 87.8% and a specificity (Spe) of 86% on the same independent test [17]. On the basis of these early studies, many researchers have designed different hybrid feature representation models to help boost the recognition capability of AOPs, including AOPs-SVM [18], SeqSVM [19], Vote9 [9], and IDAod [20]. In addition, several feature selection techniques were adopted to reduce the irrelevant and noisy features and thus enhance the predictive Acc of AOPs [21–26]. More details can be seen in the recent review article [12].

The article "Accurate Identification of Antioxidant Proteins Based on a Combination of Machine Learning Techniques and Hidden Markov Model Profiles" was published in 2021. Journal: Comput Math Methods Med.

Previous studies have shown that the hidden Markov model (HMM) profiles generated by running the HHblits [27] program can provide important clues for many protein classification tasks such as DNA-binding protein prediction [28–30] and protein fold recognition [31], similar to PSSM profiles. In general, the HMM of a query protein is an *L* × 30 matrix calculated by using the HHblits [27] software package to iteratively search a given protein against a specified database to detect its distantly related homologous proteins above a specified e-value score, where *L* is the length of the query sequence. To the best of our knowledge, there is no published paper on the application of HMM profiles in the identification of AOPs. In this study, we proposed a novel method, called AOP-HMM, which explored evolutionary features from the HMM profiles to predict AOPs. The workflow diagram of the AOP-HMM model is illustrated in Figure 1. First, three feature extraction schemes were applied to transform HMM profiles into fixed-length numerical vectors, including AAC, DPC, and auto cross-covariance (ACC) variables. Next, the optimal ACC features were selected by the ANOVA method and input to an SVM classifier to perform the prediction of AOPs. Then, the synthetic minority oversampling technique (SMOTE) [32] was adopted to deal with the unbalanced data. Finally, the proposed AOP-HMM model was validated on the two working datasets by using the 10-fold cross-validation (CV), the jackknife test, and the independent test, respectively. The experimental results showed that AOP-HMM achieved promising prediction performance and could be used in combination with existing tools to help increase annotation levels of AOPs.

## 2. Materials and Methods

### 2.1. Datasets

The construction of a high-quality benchmark dataset is the prerequisite step in developing and validating machine learning models for the identification of AOPs. In this study, two well-established datasets were adopted to examine the performance of the proposed method, denoted by D1 and D2. The D1 dataset contains 253 AOPs and 1552 non-AOPs, which was constructed by Feng et al. [14, 15] according to the following three rigorous criteria: (1) only proteins with the experimentally validated antioxidant activity were collected from the UniProt database [33]; (2) proteins with unknown residues, such as “X”, “Z”, or “B”, were excluded due to their indeterminate meanings; and (3) those proteins that have more than 60% sequence identity with any other sequences were eliminated. Based on the D1 dataset, our model was tested by using the 10-fold CV and the jackknife CV.

The article "Accurate Identification of Antioxidant Proteins Based on a Combination of Machine Learning Techniques and Hidden Markov Model Profiles" was published in 2021. Journal: Comput Math Methods Med.

Additionally, the D2 dataset provided by Zhang et al. [17] was further applied to evaluate the robustness and generalization ability of our predictor. This dataset consists of two parts: the first one contains 100 AOPs and 100 non-AOPs (termed D2_train); and the other one includes 74 AOPs and 392 non-AOPs (termed D2_test), which was adopted for the independent test.

### 2.2. Feature Extraction

#### 2.2.1. HMM Profiles

The increasing studies have shown that HMM profiles could provide informative evolutionary features for a range of protein classification tasks such as protein fold recognition [31], protein remote homology detection [34], DNA-binding protein identification [28, 29], and nucleic-acid-binding residue recognition [35]. For a query protein with the length of *L*, the HHblits program [27] was used to search against the latest Uniclust30 database [36] with default parameters to generate an HMM matrix with the size of *L* × 30. Similar to the PSSM profile, we only used the first 20 columns which represent observed frequencies for 20 natural amino acids in homologous sequences at each position. Each element *x* of the HMM profile was transformed into the range of [0,1] using the following formula:

(1) $$\begin{array}{c} f\left(x\right)=\left\{\begin{array}{cc} 0, & \text{if }x=*,\\ \;2^{-x/1000}, & \text{else}. \end{array}\right. \end{array}$$

#### 2.2.2. Composition-Based Features

The amino acid composition (AAC) of a protein is one of the most simple and effective feature representation models due to its close relation to function properties of the protein. AAC features count the frequencies of individual amino acids in the protein sequence, which can be calculated based on the sequence itself or its HMM profile, denoted by Seq-AAC and HMM-AAC.

Given a query protein sequence *S* with the length of *L*, we denote its standardized HMM matrix as *H* = [*h*_*i*,*j*_]. To help clarify the relationship between Seq-AAC and HMM-AAC, the 20 amino acids are first represented as 20 binary vectors by the one-hot encoding. For instance, the *j*th amino acid *A*_*j*_ is encoded as (0, 0,…, 1, 0,…, 0), where only the *j*th value is 1. Accordingly, a query sequence *S* is denoted as a binary matrix *B* = [*b*_*i*,*j*_], which has the same dimension with *H* = [*h*_*i*,*j*_].

The article "Accurate Identification of Antioxidant Proteins Based on a Combination of Machine Learning Techniques and Hidden Markov Model Profiles" was published in 2021. Journal: Comput Math Methods Med.

Then, the frequency of amino acid *A*_*j*_ in the query sequence *S* can be computed as

(2) $$\begin{array}{c} x_{j}=\frac{1}{L}\overset{L}{\underset{i=1}{\sum }}b_{i,j}\left(j=1,2,\cdots ,20\right). \end{array}$$

Finally, the Seq-AAC descriptor of the query sequence *S* is a 20D vector, denoted by

(3) $$\begin{array}{c} X=\left(x_{1},x_{2},\cdots ,x_{20}\right). \end{array}$$

Similarly, the HMM-AAC features can be calculated based on the HMM matrix *H* = [*h*_*i*,*j*_] instead of the binary matrix *B* = [*b*_*i*,*j*_].

At the same time, the dipeptide composition (DPC) provides more features since they may partially reflect the local sequence-order information between amino acid pairs. There are two ways to generate DPC features by using the binary matrix and the HMM matrix, termed as Seq-DPC and HMM-DPC. Here, we only give the definition formula of HMM-DPC as follows:

(4) $$\begin{array}{c} Y=\left[y_{i,j}\right], \end{array}$$

where

(5) $$\begin{array}{c} y_{i,j}=\frac{1}{L-1}\overset{L-1}{\underset{k=1}{\sum }}h_{k,i}\times h_{k+1,j}\left(1\leq i,j\leq 20\right) \end{array}$$

represents the composition of amino acid pair *A*_*i*_*A*_*j*_ in the query sequence *S*.

Since there are 400 possible combinations of dipeptides, the dimensions of both Seq-DPC and HMM-DPC are 400.

#### 2.2.3. ACC Features

In this study, each column of the HMM profile can be viewed as a time series of the corresponding property. The ACC features consist of two variables, i.e., auto covariance (AC) and cross-covariance (CC). In signal processing, the AC variable measures the correlation of a time series with a delayed copy of itself as a function of delay and the CC variable is a measure of similarity of two series as a function of the displacement of one relative to the other. Particularly, the AC is treated as the CC of a signal sequence with itself. The ACC features have been successfully applied to a wide range of sequence classification tasks in bioinformatics [37–40]. They are defined by the following formulas:

(6) $$\begin{array}{c} z_{j,k,g}=\frac{1}{L-g}\overset{L-g}{\underset{i=1}{\sum }}\left(h_{i,j}-\overset{¯}{h_{j}}\right)\left(h_{i+g,k}-\overset{¯}{h_{k}}\right)\left(1\leq j,k\leq 20,1\leq g\leq G\right), \end{array}$$

where *G* is the maximum value of the lag *g* and $\overset{¯}{h_{j}}\;\left(\overset{¯}{h_{k}}\right)$ is the average score of the *j*th (*k*th) column in the HMM matrix.

Hence, the ACC descriptor of the query sequence *S* is expressed as a 3D matrix *Z* = [*z*_*j*,*k*,*g*_] with the size of 20 × 20 × *G*, resulting in 400 × *G* features. The parameter *G* should be smaller than the length of the shortest protein sequence in the dataset. Aided by the ACC transformation of the HMM profile, the sequence-order effect and evolutionary information can be indirectly and partially, but quite effectively reflected.

The article "Accurate Identification of Antioxidant Proteins Based on a Combination of Machine Learning Techniques and Hidden Markov Model Profiles" was published in 2021. Journal: Comput Math Methods Med.

### 2.3. Feature Selection

In machine learning, a high-dimensional feature space often contains redundant and noisy information and leads to huge computational cost in the process of model training. Therefore, feature selection is one of the important steps while building a machine learning model, with the goal of finding the best possible subset of relevant features. A variety of feature selection techniques have been used for the identification of AOPs [17–19] and for other classification problems in bioinformatics [41–44]. In this study, the ANOVA method was adopted to perform the feature selection due to its simplicity and efficiency. According to the principle of ANOVA, the *F*-score of each feature was first calculated based on the ratio of the sample variance between groups to the sample variance within groups. Obviously, the larger the *F*-score, the more important the feature. Then, all features were ranked according to their *F*-score values. Finally, the optimal number of features was determined by a stepwise incremental approach.

### 2.4. Classification Algorithm

In this study, the prediction of AOPs was defined as a two-group classification problem. Here, the SVM algorithm was employed as the predictor for annotating AOPs since it is regarded as one of the most robust prediction methods, especially suitable for the binary classification. First, SVM maps the training samples into a high-dimensional feature space by using the kernel trick. Then, a good separation is achieved by the optimal hyperplane which maximizes the margin between the two classes. Finally, new testing samples are mapped into the same space and predicted to belong to a category based on which side of the gap they fall. More details about the fundamentals of SVM theory can be seen in the famous literature written by Cortes and Vapnik [45].

The performance of an SVM classifier depends on the selection of the kernel and the kernel's parameters. The radial basis function (RBF) was adopted in our experiments because of its excellent efficiency. The best combination of the two parameters *C* and *γ* was selected by a grid search scheme in the ranges of {2^−3^, 2^−1^, ⋯, 2^13^, 2^15^} and {2^3^, 2^5^, ⋯, 2^−13^, 2^−15^}.

### 2.5. SMOTE

The working dataset used in this study is quite unbalanced, with the AOPs and the non-AOPs at a ratio of 1 : 6. This may lead to the biased prediction to the predominant target class. To solve this problem, the synthetic minority oversampling technique (SMOTE) [32] was utilized to balance the dataset before building the machine learning model. SMOTE is an oversampling technique where the synthetic samples are generated for the minority class, implemented as follows: (1) take a sample *X* from the minority class, and find its *k* nearest neighbours in the feature space; (2) take the vector *V* between the current sample *X* and one of those *k* neighbours; (3) synthesize a new sample *X*′ by multiplying the vector *V* by a random number between 0 and 1; and (4) add the new sample *X*′ to the minority class. The SMOTE algorithm will continue to execute until the dataset is balanced.

The article "Accurate Identification of Antioxidant Proteins Based on a Combination of Machine Learning Techniques and Hidden Markov Model Profiles" was published in 2021. Journal: Comput Math Methods Med.

### 2.6. Performance Measurement

The proposed model was rigorously and fairly examined based on the 10-fold CV, the jackknife CV, and the independent test, respectively. The four common performance measurements were reported, including sensitivity (Sen), specificity (Spe), accuracy (Acc), and Matthews correlation coefficient (MCC). They are defined as follows:

(7) $$\begin{array}{c} \text{Sen}=\frac{\text{TP}}{\text{TP}+\text{FN}},\\ \text{Spe}=\frac{\text{TN}}{\text{TN}+\text{FP}},\\ \text{Acc}=\frac{\text{TP}+\text{TN}}{\text{TP}+\text{FP}+\text{TN}+\text{FN}},\\ \text{MCC}=\frac{\left(\text{TP}\times \text{TN}\right)-\left(\text{FN}\times \text{FP}\right)}{\sqrt{\left(\text{TP}+\text{FN}\right)\times \left(\text{TN}+\text{FP}\right)\times \left(\text{TP}+\text{FP}\right)\times \left(\text{TN}+\text{FN}\right)}}, \end{array}$$

where FP, FN, TP, and TN indicate the numbers of false positives, false negatives, true positives, and true negatives, respectively. Additionally, the value of the area under the receiver operating characteristic (ROC) curve (AUC) [46, 47] was calculated, as a reliable performance metric. In general, the larger the AUC value, the more excellent the performance of the model.

## 3. Results and Discussion

### 3.1. The Importance of Evolutionary Features Based on HMM Profiles

In this section, we employed an SVM classifier to compare the performances of HMM-based and sequence-based feature encoding models, including Seq-AAC, Seq-DPC, HMM-AAC, and HMM-DPC. All the experiments were performed on the D1 dataset by using the 10-fold CV, and five evaluation metrics are reported in Table 1. Referring to Table 1, two sequence-based models (i.e., Seq-AAC and Seq-DPC) achieved the satisfactory Spe values higher than 97% but their Sen values were lower than 40%. The HMM-DPC model together with the HMM-AAC model performed better than other sequence-based models in terms of Acc, Sen, MCC, and AUC. Particularly, the value of Sen was significantly improved from 0.2964 to 0.6324. This demonstrated that evolutionary information in the form of HMM profiles could play crucial roles in the prediction of AOPs. In addition, the performance of the HMM-AAC model was slightly inferior to that of the HMM-DPC model. This may be because the sequence-order information would be completely lost if only AAC features were used to represent the protein sequences. Hence, how to extract features related to sequence order from HMM profiles is of great importance to the annotation of AOPs.

The article "Accurate Identification of Antioxidant Proteins Based on a Combination of Machine Learning Techniques and Hidden Markov Model Profiles" was published in 2021. Journal: Comput Math Methods Med.

### 3.2. The Effect of Parameter *G*

In the AOP-HMM model, the ACC variables measure the average correlation of two amino acids separated by *g* positions along the protein sequence. Theoretically, the value of parameter *g* can be any integer between 1 and *L* − 1, where *L* is the length of the shortest sequence in the dataset. In our model, each protein sequence was represented as a 400 × *G*-dimensional (D) feature vector, where *G* was defined as the maximum value of *g*. To determine the effect of *G* on the prediction performance, we applied the SVM classifier to perform the 10-fold CV on the D1 dataset with different values of *G*. The Acc and MCC were adopted as the evaluation indicators, and the comparison results are illustrated in Figure 2. As can be seen, the values of Acc and MCC tended to stabilize with the growth of *G* and the best ones were obtained when *G* = 10. Given that too large *G* may cause the curse of dimensionality, the optimal value of *G* was set to 10 for the further study.

### 3.3. Model Optimization

There existed two thorny problems in the proposed AOP-HMM model: one is the too high dimension of feature space, and the other is the imbalance of sample sizes between AOPs and non-AOPs. In this section, we first adopted the ANOVA method to rank the total 4000 features according to their classification ability. Then, the optimal 305D features were selected to represent protein samples by using a stepwise incremental method. Finally, the SMOTE technique was applied to balance the training dataset by creating synthetic minority class examples. To evaluate the performance of model optimization, the 10-fold CV in combination with the SVM algorithm was tested on the D1 dataset. The experimental results are presented in Figure 3.

As seen in Figure 3, the SVM model with the original 4000D ACC features achieved the relatively satisfying Acc (0.946), Spe (0.994), and AUC (0.904) values, which may be attributed to the efficient utilization of sequence-order and evolutionary information by the ACC transformation. In addition, when only the selected 305D features by using the ANOVA method were used to train the SVM model, the acceptable predictive performance was obtained in comparison with that of the ACC-based model. That made sense because the dimension of feature space was dramatically reduced without much loss of Acc. However, two models based on ACC and ACC+ANOVA yielded really poor Sen (less than 0.66) and MCC (less than 0.76) values due to the unbalanced sample sizes between AOPs and non-AOPs. As expected, the ensemble model showed the best performance in terms of Acc (0.98), Sen (0.981), MCC (0.959), and AUC (0.992) and achieved the reasonable Spe (0.978) value, benefited from fusing three techniques, i.e., ACC, ANOVA, and SMOTE. Besides, ROC curves associated with three models are plotted in Figure 4, which illustrated the consistent conclusions with Figure 3.

The article "Accurate Identification of Antioxidant Proteins Based on a Combination of Machine Learning Techniques and Hidden Markov Model Profiles" was published in 2021. Journal: Comput Math Methods Med.

### 3.4. Comparison with Existing Methods

Generally speaking, the performance comparisons among different AOP prediction approaches are scientifically meaningful only if these models are trained and tested on the same datasets. For a fair comparison with the existing state-of-the-art methods, we performed the jackknife test on the D1 dataset as done in previous studies to validate the effectiveness of the proposed AOP-HMM model.  Table 2 summarized the comparison results between our method and several earlier predictors on the same dataset, including Naïve Bayes [14], AodPred [15], iANOP-Enble [48], SeqSVM [19], IDAod [20], AOPs-SVM [18], Vote9 [9], random forest [23], and hybrid feature [24].

Referring to Table 2, the proposed AOP-HMM predictor outperformed the listed state-of-the-art methods for the identification of AOPs in terms of Sen (98.23%), Acc (98.01%), MCC (0.9601), and AUC (0.992). Three models (i.e., IDAod, AOPs-SVM, and Vote9) achieved the excellent Spe values higher than 98%, but their MCC values were less than 0.75, which indicated a tendency to generate more false negatives. It is also worth noting that the IDAod tool yielded the second best Acc (97.05%) value, which automatically extracted more discriminative features from the raw *g*-gap dipeptide features by utilizing a deep autoencoder and full connect neural network. That suggested that the deep learning technique may become a practical tool in the prediction of AOPs. In addition, the AOPs-SVM classifier obtained the reasonable Acc (94.2%) and AUC (0.832) by extracting 176D discrete features composed of evolutionary information in the form of PSSM profiles and secondary structure information. This demonstrated that evolutionary features indeed help improve the performance of AOP prediction and HMM profiles could provide a useful source of evolutionary information as well as PSSM profiles.

The article "Accurate Identification of Antioxidant Proteins Based on a Combination of Machine Learning Techniques and Hidden Markov Model Profiles" was published in 2021. Journal: Comput Math Methods Med.

To further examine the robustness of the AOP-HMM model, we performed the same independent test on the D2 dataset built by Zhang et al. [16, 17]. The D2 dataset consists of two parts: (1) D2_train, including 100 AOPs and 100 non-AOPs; and (2) D2_test, including 74 AOPs and 392 non-AOPs. For the objective and unbiased assessment, the AOP-HMM was beforehand trained on the D2_train dataset and then tested on the D2_test dataset. The experimental results of our method and three previous models are reported in Table 3. The proposed method provided the highest Spe (99.5%), Acc (98.1%), MCC (0.926), and AUC (0.970) among these existing models. Additionally, the Sen of AOP-HMM was 90.5%, slightly less than that of Ahmad et al.'s method [49]. It should be pointed out that Ahmad et al. adopted three types of features, i.e., k-spaced amino acid pairs, bigram PSSM, and DPC, to train the SVM classifier. This observation reconfirmed that evolutionary features extracted from PSSM profiles or HMM profiles could play important roles in the recognition of AOPs.

From the above comparisons, the proposed method showed the impressive improvements for annotating AOPs based on the jackknife CV as well as the independent test. This may be attributed to the fusion of three techniques: (1) ACC evolutionary features extracted from HMM profiles, (2) ANOVA feature selection, and (3) SMOTE.

## 4. Conclusions

In this study, we explored a novel effective model to distinguish AOPs from non-AOPs based on a combination of machine learning techniques (ACC + ANOVA + SMOTE + SVM). Firstly, the ACC transformation was used to extract evolutionary features from HMM profiles. Secondly, the ANOVA method was performed to select the optimal feature subset by removing the redundant and noisy features. Thirdly, the SMOTE technique was utilized to oversample the imbalanced datasets. Fourthly, the SVM classifier was adopted to perform the prediction of AOPs. Finally, the 10-fold CV, the jackknife CV, and the independent test were carried out to comprehensively evaluate the performance of the proposed method, respectively. Compared with the existing state-of-the-art predictors, our method achieved superior performance and could serve as a useful tool for the automatic annotation of AOPs solely based on the sequence information. Besides, it is anticipated that the prediction ability of our model would be further enhanced by extracting hybrid features from sequences, physicochemical properties, and evolutionary information and designing powerful ensemble algorithms.

## Figures and Tables

**Figure 1:** Flowchart of the proposed AOP-HMM model.

**Figure 2:** The performance of the AOP-HMM model with different *G* values.

The article "Accurate Identification of Antioxidant Proteins Based on a Combination of Machine Learning Techniques and Hidden Markov Model Profiles" was published in 2021. Journal: Comput Math Methods Med.

**Figure 3:** The comparison results of model optimization.

**Figure 4:** ROC curves of ACC, ACC+ANOVA, and ACC+ANOVA+SMOTE models based on the 10-fold CV tests.

**Table 1:** Performance comparison between sequence-based models and HMM-based models.

Method	Acc	Sen	Spe	MCC	AUC
Seq-AAC	0.8886	0.3755	0.9722	0.4548	0.8278
Seq-DPC	0.8975	0.2964	0.9955	0.4867	0.8225
HMM-AAC	0.9296	0.5454	0.9922	0.6763	0.8579
HMM-DPC	0.9335	0.6324	0.9826	0.7006	0.9025

**Table 2:** Performance comparisons on the D1 dataset.

Methods	Sen (%)	Spe (%)	Acc (%)	MCC	AUC
Naïve Bayes [14]	72.04	66.05	66.88	—	0.855
AodPred [15]	75.09	74.48	74.79	—	—
iANOP-Enble [48]	72.78	90.75	88.25	0.5725	0.935
SeqSVM [19]	—	—	89.46	—	—
IDAod3 [20]	81.27	99.59	97.05	0.7409	—
AOPs-SVM [18]	68.0	98.5	94.2	0.741	0.832
Vote9 [9]	66.4	98.6	94.1	0.740	—
Random forest [23]	81.5	85.1	84.6	—	—
Hybrid feature [24]	66.50	96.30	83.91	—	—
AOP-HMM	98.23	97.78	98.01	0.9601	0.992

Note: results of iANOP-Enble and random forest were obtained by performing the 10-fold CV.

**Table 3:** Performance comparisons on the D2 independent dataset.

Methods	Sen (%)	Spe (%)	Acc (%)	MCC	AUC
Zhang2015 [16]	91	79	81	0.54	0.94
Zhang2016 [17]	87.8	86.0	86.3	0.617	0.948
Ahmad2020 [49]	94.14	88.15	93.71	0.92	—
AOP-HMM	90.5	99.5	98.1	0.926	0.970

## Data Availability

The data used to support the findings of this study are freely available to the academic community at https://github.com/taigangliu/AOP-HMM.
